# Chemical Speciation and Potential Mobility of Heavy Metals in the Soil of Former Tin Mining Catchment

**DOI:** 10.1100/2012/125608

**Published:** 2012-04-01

**Authors:** M. A. Ashraf, M. J. Maah, I. Yusoff

**Affiliations:** ^1^Department of Chemistry, University of Malaya, 50603 Kuala Lumpur, Malaysia; ^2^Department of Geology, University of Malaya, 50603 Kuala Lumpur, Malaysia

## Abstract

This study describes the chemical speciation of Pb, Zn, Cu, Cr, As, and Sn in soil of former tin mining catchment. Total five sites were selected for sampling and subsequent subsamples were collected from each site in order to create a composite sample for analysis. Samples were analysed by the sequential extraction procedure using optical emission spectrometry (ICP OES). Small amounts of Cu, Cr, and As retrieved from the exchangeable phase, the ready available for biogeochemical cycles in the ecosystem. Low quantities of Cu and As could be taken up by plants in these kind of acidic soils. Zn not detected in the bioavailable forms while Pb is only present in negligible amounts in very few samples. The absence of mobile forms of Pb eliminates the toxic risk both in the trophic chain and its migration downwards the soil profile. The results also indicate that most of the metals have high abundance in residual fraction indicating lithogenic origin and low bioavailability of the metals in the studied soil. The average potential mobility for the metals giving the following order: Sn > Cu > Zn > Pb > Cr > As.

## 1. Introduction

Within the terrestrial ecosystem, soils play a major role in element cycling and accumulate heavy metals in concentration orders of magnitude higher than in water and air. Meanwhile, soils are the reservoir for many harmful constituents, elemental and biological, including heavy metals and trace metals, henceforth referred to as just metals [1]. Total metal content of soils is useful for many geochemical applications but often the speciation (bioavailability) of these metals is more of an interest agriculturally in terms of what is biologically extractable [2]. Speciation is defined as the identification and quantification of the different, defined species, forms, or phases in which an element occurs [3] and is essentially a function of the mineralogy and chemistry of the soil sample examined [4]. Quantification is typically done using chemical solutions of varying but specific strengths and reactivity to release metals from the different fractions of the examined soil [5]. In terms of bioavailability, various species of metals are more biologically available in the ecosystem [6]. Bioavailability and the mobility of metals are also related to each other, then higher the concentration of mobile toxic metals (Cu, Pb, Cd, and Al) in the soil column which increases the potential for plant uptake, and animal/human consumption [3, 7, 8].

Heavy metals take part in biogeochemical cycles and are not permanently fixed in soils; therefore, assessment of their distribution in soils is a key issue in many environmental studies [9]. Heavy metals are included in soil minerals as well as bound to different phases of soil particles by a variety of mechanisms, mainly absorption, ion exchange, coprecipitation, and complexation. Moreover, soil properties such as contents of organic matter, carbonates, oxides as well as soil structure and profile development influence the heavy metal mobility [10]. The knowledge of the binding of metals with the different soil phases and components is of major interest to assess the connections with other biotic and abiotic elements of the environment [11]. Nevertheless, as Cabral and Lefebvre indicate, the metal speciation is a more complex task that determination of total metal contents [12].

It is widely recognized that to assess the environmental impact of soil pollution, the determination of the metal speciation will give more information about the potential for release of contaminants and further derived processes of migration and toxicity [13, 14]. Therefore, in geo-environmental studies of risk assessment, chemical partitioning among the various geochemical phases is more useful than measurements of total heavy metals contents [15, 16]. Among the procedures to determine element speciation, those based on sequential extraction are the most widely used [14]. These works are of interest in environmental studies to inform on the interactions with other components of the biosphere as well as to outline areas of potential toxicity and to provide information on the soil micronutrient levels for agricultural use [17]. To assess the binding of heavy metals to the main fractions in soils, a five-step sequential extraction procedure based on the capacity of some extracting reagents to remove the heavy metals retained from the geochemical phases has been used [4].

It is generally recognized that information about the physio-chemical forms of the elements is required for understanding their mobility, pathways, and bioavailability. Therefore, identification and quantification of the different species or forms of phases in which the heavy metals occur is very important to determine their bioavailability in the environment.

## 2. Study Area

Bestari Jaya catchment is located at 3° 24′ 40.41′′ N and 101° 24′ 56.23′′ E. It is a part of Kuala Selangor district, located in Selangor, biggest state of the country. District Kuala Selangor has three main towns, namely, Mukim Batang Berjuntai, Mukim Ulu Tinggi, and Mukim Tanjung Karang. Bestari Jaya is located in Mukim Batang Berjuntai. Tin mining activities has ceased from last ten years, now sand mining. The catchment has total of 442 small and big mining lakes and ponds. Bestari Jaya has a tropical humid climate, with very little variations in temperature throughout the year. The average temperature of the area is 32°C during day and 23°C at night [18].

## 3. Material and Methods

### 3.1. Soil Sampling

Five sampling sites were selected in the catchment according to their edaphic characteristics to conduct this study (Figure 1). Edaphic is a nature-related to soil. Edaphic qualities may characterize the soil itself, including drainage, texture, or chemical properties such as pH [19]. To obtain a representative average sample for each site, a total of 5 samples composed from 25 subsamples were collected at each site. Samples were extracted till an average depth of 45 cm by using an automatic core driller [20].

### 3.2. Soil Analysis

The composite samples of soil were air-dried and milled so as to pass through a 2 mm sieve, homogenized and stored in plastic bags prior to laboratory analysis. The pH was measured in a 1 : 2.5 soil/H_2_O suspension using a waterproof pH/ORP meter [21]. Cation Exchange Capacity (CEC) was measured following the standard procedure [22] and the texture was analyzed by the hydrometer method as described by Gee and Bauder [23]. Organic matter was determined by the Walkley and Black procedure [6]. All parameters were determined in triplicate. For the analysis of metals homogenised soil samples were ashed in a muffle furnace at 400°C for 1 hour and were digested by microwave assisted acid digestion [24]. Solutions from digested soil samples were stored in 100 mL high-density polyethylene samples bottles at 4°C until analysis. Speciation analysis was done through sequential extraction procedure on 1 g soil by using inductively coupled plasma optical emission spectrometry ICP-OES (Varian) (Perkin Elmer AA Analyst) [4]. Concentrations, obtained after three measurements per element, are expressed in mg/kg. Working standards for chemical analyses were prepared from Perkin-Elmer stock solutions.

### 3.3. Sequential Extraction Procedure

The Tessier procedure was selected because it is well documented, widely used [4], and it has been adapted to the study of soils and dusts [25]. Therefore, this five-step procedure allows comparison of the results obtained. Problems such as variability in extraction efficiency, inaccuracy in differentiation among geochemical phases and overlapping of the chemical partitioning between the different extraction steps are well known and they have been widely reported in the literature [14, 26]. Nevertheless, usefulness of the sequential procedure to inform about the relative bonding of metals in different solid phases and therefore the forms likely to be released in the soil solution under different environmental conditions is widely recognized [27, 28].

Following the sequential extraction procedure of Tessier, the chemical partitioning of heavy metals allows to distinguish five fractions [4] representing the following chemical phases: exchangeable metals, bound to carbonates, bound to Fe–Mn oxides, bound to sulphides and organic matter and residual fraction. The procedure was carried out with an initial weight of 1 g of the sieved dry soil sample. Deionized water was used in preparing stock solutions and for each step of the leaching procedure that was obtained from a Millipore Milli-Q plus system.

To check the results of the sequential extraction, the sum of the different fractions for each element was compared with the results obtained from the total digestion. The recovery rates were very good for iron and chromium (around 95%), whereas lower recovery rates (65–80%) were obtained for zinc and manganese. As quality control, duplicate analyses as well as analyses at an external laboratory were performed on five selected samples. The sequential extraction procedure is next described.

**Fraction 1—Exchangeable Fraction**

Samples (1 g) of soil were extracted at room temperature for 1 hour with 16 mL of magnesium chloride solution (1 M MgCl_2_) at pH 7. Soil and extraction solution were thoroughly agitated throughout the extraction. This is mainly an adsorption-desorption process. Metals extracted in the exchangeable fraction include weakly adsorbed metals and can be released by ion-exchange process. Changes in the ionic composition of the water would strongly influence the ionic exchange process of metal ions with the major constituents of the samples like clays, hydrated oxides of iron, and manganese [29]. The extracted metals were then decanted from the residual soil.

**Fraction 2—Bound to Carbonates**

The metals bound to carbonate phase are affected by ion exchange and changes of pH. The residue of Fraction 1 was extracted with 16 mL of 1 M sodium acetate/acetic acid buffer at pH 5 for 5 hours at room temperature. Significant amount of trace metals can be coprecipitated with carbonates at the appropriate pH. The extracted metal solution was decanted from the residual soil. The residual soil was used for the next extraction.

**Fraction 3—Bound to Oxides**

The residue from fraction 2 was extracted under mild reducing conditions. 13.9 g of hydroxyl amine hydrochloride (NH_2_OH·HCl) was dissolved in 500 mL of distilled water to prepare 0.4 M NH_2_OH·HCl. The residue was extracted with 20 mL of 0.4 M NH_2_OH·HCl in 25% (v/v) acetic acid with agitation at 96°C in a water bath for 6 hours. Iron and manganese oxides which can be present between particles or coatings on particles are excellent substrates with large surface areas for absorbing trace metals. Under reducing conditions, Fe (III) and Mn (IV) could release adsorbed trace metals. The extracted metal solution was decanted from the residual soil which was used for the next extraction.

**Fraction 4—Bound to Organics**

The residue from fraction 3 was oxidized as follows: 3 mL of 0.02 M HNO_3_ and 5 mL of 30% (v/v) hydrogen peroxide, which has been adjusted to pH 2, was added to the residue from fraction 3. The mixture was heated to 85°C in a water bath for 2 hours with occasional agitation and allowed to cool down. Another 3 mL of 30% hydrogen peroxide, adjusted to pH 2 with HNO_3_, was then added. The mixture was heated again at 85°C for 3 h with occasional agitation and allowed to cool down. Then 5 mL of 3.2 M ammonium acetate in 20% (v/v) nitric acid was added, followed by dilution to a final volume of 20 mL with de-ionized water. Trace metals may be bound by various forms of organic matter, living organisms, and coating on mineral particles through complexation or bioaccumulation. These substances may be degraded by oxidation leading to a release of soluble metals. The extracted metal solution was decanted from the residual soil which was used for the next extraction.

**Fraction 5—Residual or Inert Fraction**

Residue from Fraction 4 was oven dried at 105°C. Digestion was carried out with a mixture of 5 mL conc. HNO_3 _(HNO_3_, 70% w/w), 10 mL of hydrofluoric acid (HF, 40% w/w) and 10 mL of perchloric acid (HClO_4_, 60% w/w) in Teflon beakers. Fraction 5 largely consists of mineral compounds, where metals are firmly bonded within crystal structure of the minerals comprising the soil. To validate the procedure, the instrument was programmed and it carried out metal detection by displaying three absorbance readings and what was reported was the average. Blanks were also used for correction of background and other sources of error. Apart from calibration before use, quality checks were also performed on the instrument by checking the absorbance after every ten sample runs.

### 3.4. Quality Assurance of Data

In order to verify the accuracy of the sequential extraction method, certified soil reference material CRM027-050 Certified Material (Resource Technology Corporation, USA) and was analyzed concurrently with the soil samples. Recovery of metal was 99% for tin, 97% for arsenic, 112% for copper, 108% for chromium, 99% for zinc, and 94% for lead and the coefficient of variation was between 3% and 7% when analyzed in triplicate (Table 5). An internal check on the results of the microwave extraction procedure, the sequential extraction procedure was performed by comparing the sum of the 4 steps (acid-soluble + reducible + oxidizable + residual) from the sequential extraction procedure with the total metal content from the microwave-assisted acid digestion procedure (Table 5). The recovery of the sequential extraction procedure was calculated as follows:

(1) $$\begin{array}{cc} & \text{Recovery}\\ & =\frac{\text{Fraction}\;\text{1}+\text{Fraction}\;\text{2}+\text{Fraction}\;\text{3}+\text{Residual}\;\text{fraction}}{\;\text{Total}\;\text{digestion}}\\ & \;\times 100. \end{array}$$

## 4. Results

Morphological characteristics of the soil of Bestari Jaya are shown in (Table 1), whereas physical and chemical characteristics of the soil are shown in (Table 2). It shows mean values of the characteristics of top 45 cm of soil of the catchment. The results of the sequential extraction of soil samples conducted in August 2011 are summarized in (Tables 3 and 5). With respect to the soil reference material CRM 027-050, the results shown in (Table 5) indicate that the sums of the 4 fractions are in agreement with the total metal contents with satisfactory recoveries (94–112%). Correlations between pH, carbonate, organic matter and clay percentages and contents of Pb, Cu, Cr, Zn, As, and Sn in the five chemical phases of the sequential extraction have been established and analysed in (Table 4).  Table 6 shows the correlations between pH, carbonate, organic matter and clay percentages and contents of Pb, Cu, Cr, Zn, As, and Sn in the five chemical phases of the sequential extraction for soil samples. The percentages of metals in the fractions are represented graphically in (Figure 2) while (Figure 3) represents charts of the average potential mobility for the metals.

## 5. Discussion 

### 5.1. Characteristics of Soil

Bestari Jaya catchment has alluvium soil having alluvial tin deposits. Alluvium is loose, unconsolidated soil, which is then eroded, deposited, and reshaped by water in some form in a nonmarine setting [30]. Alluvium is typically made up of a variety of materials, including fine particles of silt and clay and larger particles of sand and gravel and often contains a good deal of organic matter. When this loose alluvial material is deposited or cemented into a lithological unit, or lithified, it would be called an alluvial deposit. Bestari Jaya has alluvial deposits containing tin ore (cassiterite) [31]. Cassiterite, also called tinstone, heavy, metallic, hard tin dioxide (SnO_2_) that is the major ore of tin. It is colourless when pure, but brown or black when iron impurities are present [32]. 

### 5.2. Morphology

Morphologically, there is no profile development in the tintailings as a whole; as such horizon differentiation is nonexistent. This is because the deposits are young and therefore not much affected by soil forming processes, as the mine ceased operation only about 10 years ago. These soils could thus be classified as Entisols [33]. Generally, the sandy deposits occur in the well-drained areas, while the slimes occur in the depressions, where the water table varies from 50–60 cm depth. During the rainy season the water table in the depressions could rise to the surface and cause flooding [34]. 

The clayey materials appear to be reddish, with colour notation of 5YR 5/6 or redder, this could be due to leaching of some iron-rich materials. In some areas, the textural composition changes with depth, especially at sites 3 and 5. At site 5 (Table 1), the top 30 cm of the deposits are clayey, but at 30–45 cm they are sandy with a sand content of more than 95%. At best, we can describe the texture of tintailings as variable both vertically and horizontally. 

### 5.3. Physical and Chemical Properties

Table 2 shows mean values of the characteristics of top 45 cm soil samples from ex-tin mining area, Bestari Jaya. pH values ranged from acidic to neutral (4.8–7.2). The pH was acidic in the location (S4-S5), while it was slightly acidic at (S1–S3). The carbonate percentages were in a broad range and the organic matter values were less than 10%. According to SISS, criteria, the soil of the location (S4-S5) mine dumps can be considered poor in organic matter [35]. The CEC represents the ability of the soils to absorb or release cations and, consequently, is an important parameter in sites contaminated by heavy metals. Organic matter and clay minerals are responsible for the CEC. CEC ranged from low 17.81 to high 26.98 cmol/kg. According to Conesa, pH and ECs are the most important factors [36] because under acidic conditions the tailings matrix will dissolve more salts [37]. Due to the moderately acidic and saline conditions of the soil, pH and ECs could be the limiting factors for plant establishment in the studied zone. At all sampling locations, the soil showed a sandy texture. Sandy substrates generally present oxidizing conditions however, in this case, the water-saturation state of soils and the flooding of sediments explained the reducing environment [31]. 

Taking the case of the sandy deposits, it is noted that the sand content is very high with values exceeding 90%. This condition results in excessive draining and intensive leaching of bases in the soil and these will be reflected in the low CEC [32]. The presence of too much sand in particular soil will slow down the process of soil structure development and as such the soil will retain a single-grain structure unless remedial steps are undertaken quickly. The slimes however are subjected to a different set of conditions. The clay content is quite high with values exceeding 40% in some cases. Currently the structure is rather massive but in time to come the structure may develop, especially if organic matter is present [33]. The development of structure is possible in the presence of clay, silt and sand in a favourable ratio. 

Generally, the pH of these soils is low with values of 6 or less. The low pH values are possibly due to the presence of high metal contents in the area. Similar results were reported for the pH of tintailings in Dengkil, Selangor, where the pH was reported to be 2.8–3.0 [38]. Low pH values may reduce the availability of the most micronutrients. This rather low pH can easily be overcome by using organic fertilizer. Continuous application of organic fertiliser can increase the pH to a more favourable level for crop growth as well as increase the organic contents of the soil [34]. 

The CEC is low in these soils even for with more than 50% clay content. The value at sites 1 and 3 17 cmol(+)/kg dry soil or less. This is related to the mineralogy, in which kaolinite, mica, and chlorite are found to be dominant in the clay fraction [32]. The CEC of these soils can probably be improved somewhat by incorporating organic matter into the soil. Organic carbon is far too low compared to normal soils under Malaysian conditions. This is somewhat related to the recent nature of the deposits which have just been exposed by the mining operation. Incorporation of organic manure (cow dung) and/or agricultural waste from the factory (POME) is considered essential to improve the organic matter content of the soils. In so doing, soil structure development is encouraged and more nutrients are added [34]. 

### 5.4. Metal Speciation of Soil

Metal chemical speciation carried out by sequential extraction of the metals is essential to the metal mobility [4]. The results (Table 3) obtained show that the amounts of heavy metals extracted from each fraction vary widely. The order of mobility of the metals considering their abundance in the fractions is: exchangeable > bound to carbonate > bound to oxides > bound to organics > residual [4]. Oxides exist as nodules and cement between particles. These oxides hold trace metals and can be mobilized under reducing and acidic conditions. The organic phase is relatively stable in nature but can be mobilized under strong oxidizing conditions due to degradation of organic matter [4, 39]. Cr is mostly abundant in exchangeable fraction in all the samples. The abundance of Cr in exchangeable phase is 07.98% while in the residual fraction the abundance was 39.24%. Abundance of Cr in other geochemical phases was very low. This means that Cr was more mobile in this environment than other metals that are mostly abundant in the remaining four geochemical phases. Zn is mostly abundant bound to oxides with abundance of 44.87% while in the residual fraction the abundance was 33.75% in the dry season and 34.37% in the rainy season. Abundance of Zn in other fractions was low. Zn in this environment was more mobile than the metals that were mostly abundant in the Residual fraction. This is in agreement with Zerbe et al. [40]. Copper can easily complex with organic matters because of high formation of organic-Cu compounds [39]. The result of sequential extraction shows that Cu is mostly abundant (51.33%) in the fraction bound to organics. The abundance of Cu in residual fraction was 28.34%. Heavy metals with high abundance in the phase bound to organics are more available than heavy metals in the residual fraction. The remaining heavy metals, as shown in (Figure 2) had the highest abundance in the residual fraction as follows: Cd—67.32%; Pb—95.63%; Sn—36.87%; Fe—67.73%. This agrees with Ramirez et al., 2005, who reported that Cd, Fe, Mn, Ni, and Pb were mostly associated with the residual phase [41]. The results of the sequential extraction show that most of Cr, Fe, and Zn are strongly retained in the residual phase in all soils. These heavy metals are contained in the crystal lattices of minerals with strong bindings and consequently they will not be released into the environment. In the case of Mn, its higher proportion (80%) is associated to oxides and carbonates and only in the case of a change in the redox conditions towards reductive ones, Mn would be released from oxides and if conditions became acidic, it would be released from carbonates. Therefore, such changes could only be expected from an anthropogenic impact. Metals present in the residual fraction are a measure of the degree of environmental pollution. The higher the metals present in this fraction, the lower the degree of pollution [42]. Sum of concentrations of metals in different geochemical phases can be used to express the potential mobility of metals. The potential mobility of a metal can be assessed by adding up the results of the exchangeable phase, carbonate phase, oxide, and organic phase of that metal [39]. As shown in (Figure 3), the potential mobility of Cr in soil was 63.25%. The exchangeable phase represents the mobile and bioavailable heavy metal fraction. In this phase, the heavy metals have the more labile bounds and can be easily released into the environment. The presence of heavy metals in this phase where they can be taken up by plants from the soils is the most hazardous to the ecosystem. In our soils, only little Fe, Mn, and insignificant amounts of Zn detected in four soils are present in this phase. From the result of the sequential extraction in all the soil samples studied, Cr was mostly abundant in the exchangeable fraction and the abundance was lower in the residual fraction. Low abundance of a metal in the residual phase compared with its abundance in other geochemical phases indicates higher mobility of the metal in the environment. This shows that Cr would easily be released to the environment and highly toxic. High abundance of Zn bound to oxides accounts for the high potential mobility of Zn (66.25%) (Figure 3). Cu has the highest potential mobility (71.66%) of all the heavy metals due to higher decomposition and decay of organic matter, therefore, high formation of organic-Cu compounds. The potential mobility of heavy metals with high abundance in residual fraction were: Cr 32.68%; Pb 24.37%; Cu 21.44%, Zn 27.03%; As 15.10%; Sn 63.13%. These values were low compared with the values obtained for heavy metals that were more abundant in other geochemical phases. 

According to Jones and Jarvis, 1981, processes of metal mobilization-immobilization are affected by a variety of soil properties [43]. To examine this influence, correlations between pH, carbonate, organic matter and clay percentages and contents of Pb, Cu, Cr, Zn, As, and Sn in the five chemical phases of the sequential extraction have been established for all soils. As can be seen in (Table 4), apart from Cr associated with the organic phase, no significant correlations between the carbonate contents and the heavy metals were found. Between pH and the heavy metals, the only significant relationships are the positive correlation with Fe from the carbonate phase and the negative one with Fe from the organic phase. Zinc from the exchangeable phase and Mn and Cr both from the organic phase are positively related to organic matter. Iron and Cr from the organic phase are also positively related to clay contents. Although the size of data set does not allow for better results, in general the main trends reported in the literature, such as positive correlations with organic matter and clays have also been observed in our soils [44, 45]. 

### 5.5. Potential Mobility of Heavy Metals in Soil

Average potential mobility of the heavy metals in the soil is shown in (Table 6). It is also shown graphically in (Figure 3). The average potential mobility of Cr was 64.84%. High potential mobility indicates high reduction in concentration soil. Zn is mostly abundant bound to oxides and the average potential mobility of Zn was 65.94%. Under reducing and acidic conditions, Zn will easily be mobilized to the environment. Therefore compared with other metals that were mostly abundant in the residue fraction Zn was more available and toxic in the environment. The average potential mobility of Cu is 61.86%. Under strong oxidizing conditions, due to degradation of organic matter, Cu becomes very available and toxic in the environment. More metals were present in this fraction than in the other fractions which show that the degree of pollution in the environment is presently low. Pb had the least Average potential mobility (28.08%). Change in concentration was low because Pb in soil in this environment was relatively immobile. 

From Table 6 and Figure 3, the order of average potential mobility for soil agrees with the percentage reduction in concentration. High-average potential mobility indicates high percentage reduction in concentration. However, values of the percentage reduction in concentration for metals sometimes might be controlled not only by its speciation, changes in pH and salinity, but also by unknown factors [39]. Metals with anthropogenic origin are mainly extracted in the first step of sequential extraction procedures while lithogenic metals are found in the last step of the process corresponding to the residual fraction [41]. Metals at Bestari Jaya catchment, from the results of sequential extraction, were mostly anthropogenic origin due to mining activities. Analyzed heavy metals such as Pb, Cu, Cr, Zn, As, and Sn were highly abundant in the residue, implying that they were not derived from anthropogenic sources. The Bestari Jaya catchment was also subjected to heavy metal analysis and was found to contain high concentrations of Sn, As, Pb, and Zn due to anthropogenic sources such as mining activities and forest cultivation [46]. 

## 6. Conclusion

The ex-mining land of Bestari Jaya can be classified into sandy, clayey (slime), and a mixture of sandy and clayey deposits. The sandy deposit occurs in the well-drained areas, while the slime occurs in the poorly drained areas. These soils contain low amounts of bases, phosphorus, nitrogen, and organic carbon. The pH and CEC are also low. This study served to evaluate the distribution, retention, and release of Pb, Cu, Cr, Zn, As, and Sn in the selected soils of the former tin mining catchment Bestari Jaya. The results obtained from speciation studies showed that most of the metals considered had the highest abundance in the residual fraction. This indicates that the metals were immobile. The largest proportions for Pb, Cu, and Sn were extracted in the residual phase, in which metals are strongly retained in the soil minerals. This shows that soil in the environment was not likely to be polluted by these metals. Cr was found to be highly abundant in the exchangeable fraction, indicating that it could be easily released to the environment from soil. It was also likely of high toxicity in the environment. The relatively high metal content in the catchment may represent some indirect environmental risk due to clay dispersion, and disaggregated soil particles bearing heavy metals may eventually reach and accumulate in water bodies. The average potential mobility of Zn, Cu, Pb, and Sn in the soil samples studied were quite high implying that under favourable conditions they can be released to pollute the environment. The average potential mobility of the metals arranged in decreasing order was as follows: soil: Sn > Cu > Zn > Pb > Cr > As. The results of the speciation have given the present status of metal pollution and the potential pollutants in the catchment. Further research can be carried out on the speciation of heavy metals in other environmental components in the vicinity of the Bestari Jaya catchment.

## Figures and Tables

**Figure 1:** Map of Bestari Jaya catchment.

**Figure 2:** Percentages of metals in different fractions.

**Figure 3:** Potential mobility of soil.

**Table 1:** Morphological properties of the soil of Bestari Jaya catchment.

Site no.	Soil properties (August 2011)
S1	$\frac{\text{Sandy}\;\text{loam}*\text{Entisol}-10\;\text{YR}\;5/6*\text{poorly}\;\text{drained}}{\text{Sand}*\text{deep}}$
S2	$\frac{\text{clay}\;\text{loam}*\text{Entisol}-5\;\text{YR}\;5/6*\text{well}\;\text{drained}}{\text{loam}*\text{deep}}$
S3	$\frac{\text{Silty}\;\text{loam}*\text{Entisol}-10\;\text{YR}\;3/6*\text{water}\;\text{table}\;50\;\text{cm}\;}{\text{Clay}\;\text{loam}*\text{deep}}$
S4	$\frac{\text{Sand}*\text{Entisol}-10\;\text{YR}\;5/6*\text{well}\;\text{drained}}{\text{\%Sand}*\text{deep}}$
S5	$\frac{\text{Sand}*\text{Entisol}-10\;\text{YR}\;4/4*\text{water}\;\text{table}\;60\;\text{cm}\;}{\text{Flat}\;\text{silt}\;\text{clay}*\text{deep}}$

**Table 2:** Chemical and physical characteristics of soil.

Location	Sand %	Silt %	Clay %	Textural class	pH	ECs (dSm^−1^)^b^	CaCO_3_	OM^c^%	CEC (cmol(+)/kg)^d^
S1	60 ± 14	29 ± 9	11 ± 3	Sand	6.1 ± 0.02	18 ± 8	5.7 ± 0.8	8.39 ± 0.7	17.81 ± 4
S2	65 ± 13	26 ± 8	9 ± 4	Sand	6.3 ± 0.01	17 ± 7	18.4 ± 0.6	9.91 ± 0.4	19.43 ± 3
S3	67 ± 11	21 ± 9	12 ± 3	Sand	6.7 ± 0.01	11 ± 5	6.9 ± 1.2	7.98 ± 0.5	13.76 ± 3
S4	59 ± 13	30 ± 7	11 ± 2	Sand	5.1 ± 0.01	12 ± 4	12.1 ± 2.4	5.13 ± 0.3	26.98 ± 3
S5	68 ± 13	20 ± 8	12 ± 3	Sand	4.9 ± 0.01	10 ± 5	2.5 ± 0.9	4.78 ± 0.4	24.42 ± 3

± Standard deviation, *n* = 5; ^b^electrolytic conductivity; ^c^organic matter; ^d^cation exchange capacity.

**Table 3:** Heavy metals speciation in the soil.

S/N	Sample ID	Pb	Cu	Cr	Zn	As	Sn
Fraction 1: Exchangeable mg/kg (ppm)							

1	S1	03.45	02.99	03.46	02.56	01.23	12.34
2	S2	05.67	04.37	02.91	01.98	00.92	11.87
3	S3	04.34	03.76	04.23	03.67	02.11	14.17
4	S4	06.88	05.23	02.40	02.59	01.74	15.88
5	S5	03.24	04.65	03.21	03.99	00.86	12.23
	Mean	04.71	04.20	03.22	02.95	01.37	13.29
	%age	09.34%	06.44%	07.98%	09.55%	11.53%	14.64%

Fraction 2: Bound to carbonates mg/kg (ppm)							

1	S1	08.29	11.29	08.97	06.87	02.87	25.98
2	S2	11.34	08.34	09.37	05.49	03.29	28.56
3	S3	09.88	07.35	10.10	09.30	04.21	30.25
4	S4	07.78	08.34	06.56	05.34	02.39	28.99
5	S5	10.84	09.23	09.23	06.53	02.65	25.40
	Mean	09.62	08.91	08.64	06.70	03.06	27.83
	%age	18.34%	15.44%	17.98%	19.51%	27.53%	33.64%

Fraction 3: Bound to oxides mg/kg (ppm)							

1	S1	16.23	15.88	10.00	10.76	04.21	53.23
2	S2	18.29	19.24	14.21	12.34	05.53	59.65
3	S3	12.87	17.30	15.99	13.21	03.92	61.23
4	S4	19.02	11.02	16.37	10.98	05.67	58.34
5	S5	17.25	14.83	12.31	15.23	09.34	50.85
	Mean	16.73	15.65	13.77	12.50	05.73	56.61
	%age	23.76%	26.19%	24.15%	23.98%	28.21%	42.12%

Fraction 4: Bound to organics mg/kg (ppm)							

1	S1	32.14	23.56	18.91	25.88	06.72	79.34
2	S2	29.39	27.91	16.28	28.76	09.36	80.05
3	S3	24.26	30.20	23.22	34.75	10.67	68.32
4	S4	30.22	26.87	29.90	30.04	07.49	76.51
5	S5	28.95	31.64	24.24	29.80	06.99	81.49
	Mean	28.99	28.03	22.51	29.84	08.24	77.14
	%age	26.16%	28.91%	30.75%	33.58%	40.53%	52.40%

Fraction 5: Residual or inert mg/kg (ppm)							

1	S1	48.21	62.51	32.44	54.38	11.23	102.34
2	S2	52.78	70.46	21.96	78.23	14.24	098.34
3	S3	61.10	49.80	38.75	59.00	10.96	112.87
4	S4	57.91	53.77	50.02	63.22	08.34	118.34
5	S5	43.55	50.24	43.25	49.30	20.34	101.45
	Mean	52.71	57.35	37.24	60.62	13.02	106.66
	%age	57.56%	52.98%	61.45%	63.12%	59.52%	71.29%

**Table 4:** Correlation between pH, Carbonates, organic matter content, and clay percentages with contents of heavy metals (mg/kg).

Metals with fractions		pH	CO_3_^2−^	OM	Clay
			%		
Pb	Exchangeables	−0.280	0.324	0.487	0.123
	Carbonates	0.653	0.086	−0.561	−0.572
	Oxides	−0.353	−0.361	−0.235	0.183
	Organics	−0.686	0.138	0.466	0.651
	Residuals	0.141	0.282	0.077	0.096

Cu	Exchangeables	−0.223	0.558	0.221	0.246
	Carbonates	0.484	0.138	−0.348	−0.049
	Oxides	−0.331	0.268	0.530	0.278
	Organics	−0.292	0.420	0.698	0.416
	Residuals	0.408	0.085	−0.137	−0.077

Cr	Exchangeables	−0.198	0.174	0.613	0.150
	Carbonates	0.404	−0.176	−0.232	0.051
	Oxides	−0.375	−0.474	−0.037	0.251
	Organics	−0.341	0.094	0.193	0.293
	Residuals	0.243	−0.044	−0.166	−0.039

Zn	Exchangeables	−0.223	0.558	0.221	0.246
	Carbonates	0.484	0.138	−0.348	−0.049
	Oxides	−0.331	0.268	0.530	0.278
	Organics	−0.292	0.420	0.698	0.416
	Residuals	0.408	0.085	−0.137	−0.077

As	Exchangeables	−0.198	0.174	0.613	0.150
	Carbonates	0.404	−0.176	−0.232	0.051
	Oxides	−0.375	−0.474	−0.037	0.251
	Organics	−0.341	0.094	0.193	0.293
	Residuals	−0.223	0.558	0.221	0.246

Sn	Exchangables	0.484	0.138	−0.348	−0.049
	Carbonates	−0.331	0.268	0.530	0.278
	Oxides	−0.292	0.420	0.698	0.416
	Organics	0.408	0.085	−0.137	−0.077
	Residuals	−0.198	0.174	0.613	0.150

**Table 5:** Results of analysis of standard reference materials (SRM) in comparison with certified values.

Standard reference material	Analysed SRM value	Certified SRM value	Recovery%
Sequential extraction			
SRM-027-050-Soil (*n* = 3)			

Step 1			
As	4.19 ± 0.40	4.98.0 ± 0.38	88
Cr	3.13 ± 0.10	2.87 ± 0.13	85
Zn	4.08 ± 0.79	3.94 ± 0.39	100
Cu	34.24 ± 1.6	46.73 ± 1.8	69
Pb	73.11 ± 2.00	64.20 ± 2.00	101
Sn	178 ± 5.00	195 ± 2.00	103

Step 2			
As	3.08 ± 0.30	3.12 ± 0.34	90
Cr	2.89 ± 0.14	2.98 ± 0.19	85
Zn	100.18 ± 4.00	88.84 ± 3.00	92
Cu	102.38 ± 2.0	129.0 ± 2.5	101
Pb	62.30 ± 3.00	65.28 ± 3.00	99
Sn	112 ± 4.00	136 ± 5.00	100

Step 3			
As	1.18 ± 0.23	1.02 ± 0.32	95
Cr	100.12 ± 4.00	105.00 ± 5.00	106
Zn	52.28 ± 2.00	65.74 ± 3.00	103
Cu	29.28 ± 2.0	36.32 ± 2.5	100
Pb	10.10 ± 2.00	8.80 ± 3.00	102
Sn	70 ± 2.00	72 ± 3.00	100

Step 4			
As	0.18 ± 0.03	0.20 ± 0.52	120
Cr	73.33 ± 5.00	60.56 ± 4.00	128
Zn	98.00 ± 5.00	87.34 ± 4.00	120
Cu	20.98 ± 0.88	19.93 ± 2.00	115
Pb	14.23 ± 0.90	10.53 ± 1.00	104
Sn	40 ± 4.00	35 ± 2.00	111

Total digestion			
CRM-027-050-Soil (*n* = 3)			
As	9.86 ± 1.00	10.78 ± 1.00	97
Cr	157.95 ± 4.00	180.45 ± 4.00	108
Zn	251.16 ± 4.00	250.06 ± 5.00	99
Cu	198.18 ± 4.00	235.75 ± 3.00	112
Pb	143.91 ± 2.00	155.31 ± 2.00	94
Sn	390 ± 5.00	381 ± 4.00	99

**Table 6:** Analysis of heavy metals speciation.

Fraction	Description	Pb	Cu	Cr	Zn	As	Sn
1	Exchangeable	09.34%	06.44%	07.98%	09.55%	11.53%	14.64%
2	Bound to carbonates	18.34%	15.44%	17.98%	19.55%	27.53%	33.64%
3	Bound to oxides	23.76%	26.19%	24.15%	23.98%	28.21%	42.12%
4	Bound to organics	26.16%	28.91%	30.75%	33.58%	40.53%	52.40%
5	Residual or inert	57.56%	52.98%	61.45%	63.12%	59.52%	71.29%
	Sum of concentration of metals (mg/kg)	22.55	22.82	17.07	22.52	06.28	56.30
	Potential mobility	52.73%	54.88%	42.34%	52.12%	16.72%	89.14%

## References

[1] Cottenie A, Verloo M (1984). Analytical diagnosis of soil pollution with heavy metals. *Fresenius Journal of Analytical Chemistry*.

[2] Cottenie A, Camerlynck R, Verloo M, Dhaese A (1980). Fractionation and determination of trace elements in plants, soils and sediments. *Pure and Applied Chemistry*.

[3] Tack FMG, Verloo MG (1995). Chemical speciation and fractionation in soil and sediment heavy metal analysis: a review. *International Journal of Environmental Analytical Chemistry*.

[4] Tessier A, Campbell PGC, Blsson M (1979). Sequential extraction procedure for the speciation of particulate trace metals. *Analytical Chemistry*.

[5] Ryan PC, Hillier S, Wall AJ (2008). Stepwise effects of the BCR sequential chemical extraction procedure on dissolution and metal release from common ferromagnesian clay minerals: a combined solution chemistry and X-ray powder diffraction study. *Science of the Total Environment*.

[6] Nelson A, Donkin P (1985). Processes of bioaccumulation: the importance of chemical speciation. *Marine Pollution Bulletin*.

[7] Lund W (1990). Speciation analysis—why and how?. *Fresenius Journal of Analytical Chemistry*.

[8] Ratuzny T, Gong Z, Wilke BM (2009). Total concentrations and speciation of heavy metals in soils of the ShenyangZhangshi irrigation area, China. *Environmental Monitoring and Assessment*.

[9] Salim I, Miller C, Howard J Combined sequential extraction-adsorption isotherm analysis of the heavy metal retention characteristics of a michigan landfill bottom liner.

[10] Kabata-Pendias A, Pendias H (2001). *Trace elements in soils and plants*.

[11] Hirner AV (1992). Trace element speciation in soils and sediments using sequential chemical extraction methods. *International Journal of Environmental Analytical Chemistry*.

[12] Cabral AR, Lefebvre G (1998). Use of sequential extraction in the study of heavy metal retention by silty soils. *Water, Air, and Soil Pollution*.

[13] Rauret G, Rubio R, López-Sánchez JF, Casassas E (1988). Determination and speciation of copper and lead in sediments of a Mediterranean river (River Tenes, Catalonia, Spain). *Water Research*.

[14] Usero J, Gamero M, Morillo J, Gracia I (1998). Comparative study of three sequential extraction procedures for metals in marine sediments. *Environment International*.

[15] Campanella L, D’Orazio D, Petronio BM, Pietrantonio E (1995). Proposal for a metal speciation study in sediments. *Analytica Chimica Acta*.

[16] Quevauviller P, van der Sloot HA, Ure A, Muntau H, Gomez A, Rauret G (1996). Conclusions of the workshop: harmonization of leaching/extraction tests for environmental risk assessment. *Science of the Total Environment*.

[17] Wilcke W, Kretzschmar S, Bundt M, Saborío G, Zech W (1998). Aluminum and heavy metal partitioning in a horizons of soils in Costa Rican coffee plantations. *Soil Science*.

[18] Ashraf MA, Maah MJ, Yusoff I (2011). Heavy metals accumulation in plants growing in ex tin mining catchment. *International Journal of Environmental Science and Technology*.

[19] Bryson CT, Krutz LJ, Ervin GN, Reddy KN, Byrd JD (2010). Ecotype variability and edaphic characteristics for cogongrass (Imperata cylindrica) populations in Mississippi. *Invasive Plant Science and Management*.

[20] Shamshuddin J, Mokhtar N, Paramananthan S (1986). Morphology, mineralogy and chemistry of an ex-mining land in Ipoh, Perak. *Pertanika*.

[21] Thomas GW, Sparks DL (1996). Soil pH and soil acidity. *Methods for Soil Analysis. Part 3: Chemical Methods*.

[22] Rowell DJ (1994). *Soil Science, Methods and Applications*.

[23] Gee GW, Bauder JW, Klute A (1986). Particle soil analysis. *Methods for Soil Analysis. Part 1: Physical and Mineralogical Methods*.

[24] Camel V (2000). Microwave-assisted solvent extraction of environmental samples. *Trends in Analytical Chemistry*.

[25] Clevenger TE (1990). Use of sequential extraction to evaluate the heavy metals in mining wastes. *Water, Air, and Soil Pollution*.

[26] Kheboian C, Bauer CF (1987). Accuracy of selective extraction procedures for metal speciation in model aquatic sediments. *Analytical Chemistry*.

[27] Gibson MJ, Farmer JG (1986). Multi-step sequential chemical extraction of heavy metals from urban soils. *Environmental Pollution Series B*.

[28] Maskall JE, Thornton I (1998). Chemical partitioning of heavy metals in soils, clays and rocks at historical lead smelting sites. *Water, Air, and Soil Pollution*.

[29] Abu-Kukati Y (2001). Heavy metal distribution and speciation in sediments from Ziglab Dam-Jordan. *Geological Engineering*.

[30] Yilmaz I, Karacan E (1997). Geotechnical properties of alluvial soils: an example from south of Sivas (Turkey). *Bulletin of Engineering Geology and the Environment*.

[31] Petrovský E, Kapička A, Jordanova N, Borůvka L (2001). Magnetic properties of alluvial soils contaminated with lead, zinc and cadmium. *Journal of Applied Geophysics*.

[32] Gama-Castro JE, Solleiro-Rebolledo E, Vallejo-Gómez E (2000). Weathered pumice influence on selected alluvial soil properties in west Nayarit, Mexico. *Soil and Tillage Research*.

[33] Iqbal J, Thomasson JA, Jenkins JN, Owens PR, Whisler FD (2005). Spatial variability analysis of soil physical properties of alluvial soils. *Journal of Soil Science Society of America*.

[34] Shamshuddin J, Paramananthan S (1980). Acidity and charge characteristics of marine alluvial soils from Carey Islands, Selangor. *Pertanika*.

[35] SISS– Societa` Italiana per la Scienza del Suolo (1985). *Metodi Normalizzati per l’Analisi del Suolo*.

[36] Conesa HM, Faz A, Arnaldos R (2006). Heavy metal accumulation and tolerance in plants from mine tailings of the semiarid Cartagena-La Union mining district. *Science of the Total Environment*.

[37] Wong JWC, Ip CM, Wong MH (1998). Acid-forming capacity of lead-zinc mine tailings and its implications for mine rehabilitation. *Environmental Geochemistry and Health*.

[38] Maesschalk GG, Lim KH The effect of organic waste materials, fertilization and mulching on the physical properties and yield of mungbean on tin-tailings.

[39] Haung J, Haung R, Jiao JJ, Chen K (2007). Speciation and mobility of heavy metals in mud, in coastal reclamation areas in Chenzhen, China. *Environment Geology*.

[40] Zerbe J, Sobczyński T, Elbanowska H, Siepak J (1999). Speciation of heavy metals in bottom sediments of lakes. *Polish Journal of Environmental Studies*.

[41] Ramirez M, Massolo S, Frache R, Correa JA (2005). Metal speciation and environmental impact on sandy beaches due to El Salvador copper mine, Chile. *Marine Pollution Bulletin*.

[42] Howari FM, Banat KM (2001). Assessment of Fe, Zn, Cd, Hg, and Pb in the Jordan and Yarmouk River sediments in relation to their physicochemical propperties and sequential extraction characterization. *Water, Air, and Soil Pollution*.

[43] Jones LHP, Jarvis SC, Greenland DJ, Hayes MHB (1981). The fate of heavy metals. *The Chemistry of Soil Processes*.

[44] Labib FB, Khalil JB, Halaka SH (1989). Heavy metals in some soils and clay beds of Bahariya Oasis, Egypt. *Agrochimica*.

[45] Li X (1993). *The study of multielement associations in the soil—plant system in some old metalliferous mining areas*.

[46] Ashraf MA, Maah MJ, Yusoff I, Wajid A, Mahmood K (2011). Sand mining effects, causes and concerns: a case study from Bestari Jaya, Selangor, Peninsular Malaysia. *Scientific Research and Essays*.

